The article "The DnaE polymerase from Deinococcus radiodurans features RecA-dependent DNA polymerase activity" was published in 2016. Journal: Biosci Rep.

# The DnaE polymerase from *Deinococcus radiodurans* features RecA-dependent DNA polymerase activity

**DOI:** 10.1042/BSR20160364

**Published:** 2016-12-05

**Authors:** Lorenzo Randi, Alessandro Perrone, Mirko Maturi, Fabrizio Dal Piaz, Michela Camerani, Alejandro Hochkoeppler

**Affiliations:** * Department of Pharmacy and Biotechnology, University of Bologna, Viale Risorgimento 4, 40136 Bologna, Italy; † Department of Medicine, University of Salerno, Via Giovanni Paolo II, 132, 84084 Fisciano SA, Italy; ‡ CSGI, University of Firenze, Via della Lastruccia 3, 50019 Sesto Fiorentino (FI), Italy

**Keywords:** *Deinococcus radiodurans*, DnaE polymerase, DNA polymerase III, *Escherichia coli*, RecA, α subunit

## Abstract

We report in the present study on the catalytic properties of the *Deinococcus radiodurans* DNA polymerase III α subunit (αDr). The αDr enzyme was overexpressed in *Escherichia coli*, both in soluble form and as inclusion bodies. When purified from soluble protein extracts, αDr was found to be tightly associated with *E. coli* RNA polymerase, from which αDr could not be dissociated. On the contrary, when refolded from inclusion bodies, αDr was devoid of *E. coli* RNA polymerase and was purified to homogeneity. When assayed with different DNA substrates, αDr featured slower DNA extension rates when compared with the corresponding enzyme from *E. coli* (*E. coli* DNA Pol III, αEc), unless under high ionic strength conditions or in the presence of manganese. Further assays were performed using a ssDNA and a dsDNA, whose recombination yields a DNA substrate. Surprisingly, αDr was found to be incapable of recombination-dependent DNA polymerase activity, whereas αEc was competent in this action. However, in the presence of the RecA recombinase, αDr was able to efficiently extend the DNA substrate produced by recombination. Upon comparing the rates of RecA-dependent and RecA-independent DNA polymerase activities, we detected a significant activation of αDr by the recombinase. Conversely, the activity of αEc was found maximal under non-recombination conditions. Overall, our observations indicate a sharp contrast between the catalytic actions of αDr and αEc, with αDr more performing under recombination conditions, and αEc preferring DNA substrates whose extension does not require recombination events.

## Abstract (precis)

We report in the present study on the catalytic properties of *Deinococcus radiodurans* DnaE polymerase, whose DNA elongation efficiency was compared with the homologous *Escherichia coli* polymerase. Contrary to the latter, the deinococcal enzyme was found to be strictly dependent on RecA recombinase.

## INTRODUCTION

DNA polymerases (DNA Pols) are peculiar enzymes, featuring a conserved multi-domain molecular architecture. In particular, the conformation of DNA Pols resembles an open right-hand and contains three main domains, denoted by thumb, palm and fingers [1]. The thumb domain tightly associates with the double-stranded portion of the DNA substrate, whereas the 3′-OH end of the primer and the ssDNA template are allocated in the palm and in the fingers domain respectively [2]. The subsequent binding of a deoxynucleoside-triphosphate (dNTP) triggers the movement of the fingers towards the palm, poising the active site to proficient catalysis, i.e. the nucleophilic attack by the 3′-OH of the primer to the α-phosphate of the dNTP [3]. Besides this primary DNA extension activity, the complex task of genome replication demands to DNA Pols the exertion of quite a number of secondary essential functions. Among these functions, high fidelity and processive replication, as well as proper co-ordination of leading and lagging DNA strand extension, are accomplished by DNA Pol holoenzymes composed of different subunits, the assembly of which determines the actual enzyme activities [2]. *Escherichia coli* does express five distinct DNA Pols, with DNA Pol III responsible for genome replication [4–6], DNA Pol I essential for removing the multiple primers necessary for lagging strand replication [7,8] and DNA Pols II, IV and V [9–12], eventually engaged in the replication of damaged DNA. *E. coli* DNA Pol III (αEc) is composed of a catalytic core, a DnaX complex and a β-clamp. The catalytic core does contain the α, ε and θ subunits [13] respectively featuring 5′–3′ polymerase [14], 3′–5′ exonuclease (proofreading) [15] and ε-stabilizing activity [16,17]. Notably, DNA Pol III α subunit, which is coded by the *dnaE* gene, is the only essential replicase in *E. coli*. The DnaX complex contains the τ, δ, δ’, χ and Ψ subunits [18], according to a stoichiometry τ_3_δδ’χψ [19]. This complex catalyses the loading of the β-clamp on to DNA, and interacts with the core α subunit. The β-clamp is a homodimer, and confers to the holoenzyme high processivity by tethering the polymerase to the DNA substrate [20,21]. In addition, the progression of a replication fork is assisted by the association of DNA Pol III with DNA helicase and primase [22,23]. Interestingly, it was shown that β-clamp, helicase and primase are competent in interacting with *E. coli* DNA Pols II, IV and V [24], whose action is assisted by the RecA recombinase [25–27]. More recently, it was also elegantly demonstrated that RecA activates replisomes containing DNA Pol II, Pol IV or Pol V [28], and inhibits DNA Pol III holoenzyme [28]. In addition, it was observed that the overexpression of Pol IV and RecA slows down the progression of Pol III replication forks [29], suggesting that RecA inhibits the action of Pol III holoenzyme in *E. coli*.

*Deinococcus radiodurans* is a Gram-positive bacterium, belonging to the Deinococcales order, whose members feature outstanding radioresistance [30]. *D. radiodurans* was indeed first isolated from canned meat samples, exposed to γ-rays in order to obtain a sterile, and hence stable, food supply [31]. Contrary to the vast majority of prokaryotes, *D. radiodurans* cells are polyploid, with the actual ploidy number being affected by growth phase [32] and culture medium [33]. Each genome copy consists of two chromosomes (containing 2.6 and 0.4 Mbp) and two plasmids, featuring 177×10^3^ and 45.7×10^3^ bp respectively [34]. Three different DNA Pols were identified in *D. radiodurans*, i.e. DNA Pol I [35], Pol III [36] and Pol X [37], among which DNA Pol III α subunit (DnaE) is essential for viability [36,38]. Rather astonishingly, cells of *D. radiodurans* exposed to 14 kGy, and containing fragmented chromosomes, are able to reconstruct their genomes within 6–7 h after radiation exposure [30]. Although polyploidy is an obvious requisite for this genome reconstruction competence, *D. radiodurans* does also feature additional and peculiar biochemical properties responsible for genome integrity maintenance. In particular, when considering that ionizing radiations induce severe oxidative stress, it was realized that the radiation-resistance of *D. radiodurans* is mainly due to biochemical factors preserving the proteome of this bacterium from oxidation damages [30]. Nevertheless, the capability of *D. radiodurans* to reconstruct its highly fragmented genome does also imply an outstanding DNA repair competence. To accomplish this task, *D. radiodurans* first depends on RecJ, which is essential for viability [39] and features 5′–3′ exonuclease activity. The action of this enzyme produces 3′ overhangs at the expense of chromosomal/plasmid fragments, triggering the RecFOR-mediated loading of RecA on to DNA. Subsequently, the recombinase activity of RecA and the DNA polymerase activity of DnaE catalyse the recombination of overlapping homologous fragments and the extension of the recombinant molecules respectively. This mechanism, denominated extensive synthesis-dependent strand annealing (ESDSA), does progressively increase the molecular mass of DNA fragments, whose number decreases in parallel. Besides the impairment of ESDSA, both *recA* and *dnaE* mutations confer interesting phenotypes to *D. radiodurans*: (i) *ΔrecA* strains feature poor viability and extreme radiation sensitivity [39–41]; (ii) under physiological conditions (no irradiation), *recA* mutants do replicate DNA at slower rates when compared with wild-type [36]; (iii) temperature-sensitive *dnaE* mutants feature lower radiation-resistance than strains defective in DNA polymerase I (PolA) [35,36]. In particular, the poor DNA replication efficiency of unirradiated RecA^−^ strains suggests a role for this recombinase in DnaE-catalysed replication.

Both DNA Pol I and DNA Pol X from *D. radiodurans* were previously purified, and their catalytic performances were investigated [35,42–45]. On the contrary, the α subunit (DnaE) of *D. radiodurans* DNA Pol III (αDr) has never been isolated to homogeneity *in vitro*. In the present study, we report on the overexpression and purification of this enzyme, along with the characterization of its catalytic properties at the expense of different DNA substrates, in the presence or in the absence of RecA. Further, we used the well-known α subunit (DnaE) of *E. coli* DNA Pol III (here denominated αEc) as a reference polymerase, and we report on the comparison of these two enzymes, whose action is essential for their respective organisms.

## MATERIALS AND METHODS

### Bacterial strains, plasmids and growth media

*Escherichia coli* BW25993 [genotype: *Δ*(*araD-araB*)*567*, *rph-1*, *Δ*(*rhaD-rhaB*)*568*, *hsdR514*] was obtained by Mary Berlyn (*Escherichia coli* Genetic Stock Center, CGSC, Yale University), and *E. coli* TOP10 [genotype: F^−^ *mcrA* Δ(*mrr-hsdRMS-mcrBC*) ϕ80*lacZΔM15* Δ*lacX74 recA1 araD139* Δ(*ara-leu*)*7697 galU galK rpsL endA1 nupG*] was purchased from Invitrogen. Both strains were grown in LB medium (10, 10 and 5 g/l respectively, of Tryptone, NaCl and Yeast Extract), supplemented, when appropriate, with 100 μg/ml of ampicillin. The plasmid pBAD-α1160, containing an insert coding for the full-length α subunit of *E. coli* DNA Polymerase III (αEc), was previously described [46], and will be indicated here as pBAD-αEc. The gene coding for the full-length α subunit of *Deinococcus radiodurans* DNA Polymerase III (αDr) was optimized for *E. coli* codon usage and synthesized by GenScript. The synthetic gene was inserted into the pBAD-HisB plasmid, using the *Nco*I and *Pst*I sites at 5′ and 3′ ends respectively, yielding pBAD-αDr. This vector was used to transform both *E. coli* strains BW25993 and TOP10, the transformants were isolated and purified on LB Petri dishes containing 100 μg/ml of ampicillin, and then stored at −20°C in LB–glycerol (15%, v/v) medium. Proteins overexpression was triggered in LB medium by the addition of 1 mM arabinose.

### Proteins overexpression

The overexpression of αEc was performed as recently described [47]. The overexpression of soluble αDr was attempted using both *E. coli* strains TOP10 and BW25993. In *E. coli* TOP10, the target protein was expressed at low concentrations, irrespective of temperature for growth and induction length. On the contrary, the BW25993 strain did perform much better, and was used throughout to overexpress soluble αDr. In particular, single colonies of *E. coli* BW25993/pBAD-αDr were picked from LB–ampicillin Petri dishes, transferred to LB–ampicillin liquid medium and pre-cultured at 37°C for 8 h. The pre-cultures were then diluted (1:500) in fresh LB medium, grown for 15 h at 37°C, and the cultures were finally induced at 37°C for 3 h. Cells were collected by centrifugation (10000 × ***g***, 20 min, 4°C), and the pellets were stored at −20°C until used.

To overexpress αDr in the form of inclusion bodies, single colonies of *E. coli* TOP10/pBAD-αDr were pre-cultured in LB medium for 15 h at 37°C. The pre-cultures were then diluted (1:500) in fresh LB medium, grown for 8 h, and finally induced for 15 h at 37°C. After harvest, the cell pellets were stored at −20°C.

### Extraction of soluble proteins

To isolate soluble protein extracts, cells were resuspended in Buffer A, consisting of 50 mM Tris/HCl (pH 8), 50 mM NaCl, 1 mM EDTA, 2.5 mM DTT, and gently homogenized with a cold glass potter. The cell suspension was then supplemented with 1 mM PMSF and subjected to 7 cycles of sonication at 6 W. Each sonication cycle consisted of 15 s of impulse, followed by 15 s of cooling interval, for a total time of 2 min. The extracts accordingly obtained were centrifuged (10000 × ***g***, 20 min, 4°C), the pellets were discarded, and the supernatant was immediately used to purify soluble proteins.

### Solubilization of proteins from inclusion bodies

*E. coli* TOP10/pBAD-αDr cells were disrupted as described for the extraction of soluble proteins. After sonication, the extract was centrifuged at 4000 × ***g*** (20 min, 4°C), and the pellet (containing the inclusion bodies) was washed twice with 200 mM Tris/HCl (pH 8), 500 mM NaCl, 1 mM DTT, 0.1% (v/v) Triton-X-100. After the second wash, the pellet was harvested and stored at −20°C until used. To solubilize proteins, inclusion bodies were resuspended in 200 mM Tris/HCl (pH 8), 500 mM NaCl, 5 mM β-mercaptoethanol, 6 M urea, using 100 ml of buffer per g (wet weight) of sample. After incubation at room temperature for 3 h under magnetic stirring, the solution was centrifuged at 16000 × ***g*** (20 min, 20°C), and the pellet was discarded, yielding a supernatant containing 50 mg of proteins per g of inclusion bodies. To refold proteins, the supernatant was subjected to four dialysis steps, against: (i) 200 mM Tris/HCl (pH 8), 500 mM NaCl, 5 mM β-mercaptoethanol, 2 mM MgCl_2_, 4 M urea; (ii) 100 mM Tris/HCl, 500 mM NaCl, 5 mM β-mercaptoethanol, 2 mM MgCl_2_, 2 M urea; (iii) 50 mM Tris/HCl, 200 mM NaCl, 5 mM β-mercaptoethanol, 2 mM MgCl_2_, 1 M urea and (iv) 50 mM Tris/HCl, 50 mM NaCl, 5 mM β-mercaptoethanol, 2 mM MgCl_2_, 10% (v/v) glycerol. The dialysis tube contained 30 ml of sample per litre of external buffer.

### Purification of soluble proteins

The α subunit of *E. coli* DNA Pol III was purified as previously described [47], and the same procedure was used to isolate homogeneous αDr. Briefly, the soluble protein extracts were subjected to anion-exchange chromatography (Q-Sepharose FF, 50 ml column) in Buffer A, applying a linear 50–600 mM NaCl gradient. The best fractions, according to SDS/PAGE analysis, were pooled, desalted, concentrated, supplemented with 20% (v/v) glycerol, 5 mM MgCl_2_ and loaded on to a Cibacron Blue column (15 ml). After extensive washing of the column with Buffer B (Buffer A containing 20% glycerol and 5 mM MgCl_2_), αDr was eluted with the same buffer containing 1 M NaCl. The eluted peak was desalted and loaded on to a HiTrap Heparin column (5 ml), to which a linear 50–600 mM gradient of NaCl was applied. The best fractions were reconditioned to 50 mM NaCl with Buffer A containing 20% glycerol, and they were finally subjected to a second anion-exchange chromatography, using a HiTrap Q column (5 ml). The best fractions, containing partially purified αDr, were pooled and stored at −20°C until used.

### Purification of αDr from inclusion bodies

The refolded sample was loaded on to a Cibacron Blue column (15 ml), and after a washing step (six column volumes), αDr was eluted with Buffer B containing 1 M NaCl. After dialysis against Buffer A containing 20% glycerol, the sample was loaded on to a HiTrap Heparin column (5 ml) and subjected to a linear 50–600 mM NaCl gradient. The best fractions were pooled and stored at −20°C until used.

### MS

Elution of proteins from acrylamide gels, trypsin digestion and separation of peptides were performed as previously described [17]. The resulting peptides were analysed by LC-MS/MS using an Orbitrap XL instrument (Thermo Fisher Scientific) equipped with a nano-ESI source coupled with a nano-Acquity capillary UPLC (Waters). Briefly, peptides were separated with a capillary BEH C18 column (0.075×100 mm, 1.7 μM, Waters) using aqueous 0.1% formic acid (A) and CH_3_CN containing 0.1% formic acid (B) as mobile phases. Peptides were eluted by means of a linear gradient from 5 to 50% of B in 90 min, at a 300 nl/min flow rate. Mass spectra were acquired over an *m*/*z* range from 400 to 1800. To achieve protein identification, MS and MS/MS data underwent Mascot Search Engine software analysis to interrogate the National Center for Biotechnology Information nonredundant (NCBInr) protein database. Parameters sets were: trypsin cleavage; carbamidomethylation of cysteines as a fixed modification and methionine oxidation as a variable modification; a maximum of two missed cleavages; false discovery rate, calculated by searching the decoy database, 0.05.

### Enzyme assays

Type XV activated calf-thymus DNA was obtained from Sigma–Aldrich. *E. coli* RecA recombinase and dNTPs mixture (dATP, dGTP, dTTP and dCTP, 10 mM each) were purchased from NEB. Oligonucleotides, to be annealed and used as DNA substrates, were synthesized by GenScript. DNA polymerase activity was determined according to our previously described enzyme-coupled assay, which was designed for the continuous spectrophotometric detection of PP_i_/phosphate [48]. Briefly, reactions were assayed in 100 mM Tris/HCl (pH 8), 5 mM MgCl_2_, 0.25 mM inosine, 100 μM dNTPs and 10, 50 and 500 m-units/ml of inorganic pyrophosphatase (PPase), purine nucleoside phosphorylase (PNPase) and xanthine oxidase (XOD) respectively. The uric acid generated by XOD was detected at 293 nm, and phosphate concentrations were calculated assuming a molar absorption coefficient for uric acid equal to 12600 M^−1^ · cm^−1^ [49]. The ATPase activity of RecA was determined detecting both the P_i_ and the ADP generated. To continuously determine the release of ADP, the reaction mixture contained 100 mM Tris/HCl (pH 8), 10 mM MgCl_2_, 20 mM KCl, 0.5 mM phosphoenolpyruvate (PEP), 1.5 unit/ml of pyruvate kinase (PK), 0.25 mM β-NADH and 6 units/ml of lactate dehydrogenase (LDH). By this means, the ATP consumed by RecA is regenerated from ADP and PEP, which is converted to pyruvate by PK; finally, pyruvate is reduced, in the presence of β-NADH, to lactate. Reactions were monitored at 340 nm, and the molar absorption coefficient of β-NADH was assumed equal to 6200 M^−1^ · cm^−1^.

The lag time before steady-state intermediate concentrations is reached, as we observed in the present study, is well-known for enzyme coupled assays [50]. Activities were determined by considering the interval time, subsequent to the lag, during which zero-order kinetics was detected.

All the assays were performed using a Cary 300 UV–VIS spectrophotometer. Protein concentration was determined according to Bradford [51], using BSA as standard.

## RESULTS

### Overexpression of soluble *D. radiodurans* DnaE polymerase

We first attempted the overexpression of *D. radiodurans* αDr in soluble form. To this aim, we transformed *E. coli* TOP10 with pBAD-αDr, and we searched for growth and induction conditions corresponding to overexpression yields compatible with the purification of the target protein. However, using *E. coli* TOP10/pBAD-αDr we were not able to obtain satisfactory amounts of soluble αDr (results not shown). On the contrary, when *E. coli* BW25993/pBAD-αDr was grown at 37°C and induced for 3 h at the same temperature, high overexpression of soluble αDr was observed (Supplementary Figure S1A). Soluble protein extracts were accordingly prepared from this bacterial host, and the purification of αDr was pursued by four consecutive chromatographic steps (see Materials and Methods). By this means, we significantly purified αDr (Supplementary Figure S1B and Table 1), but we could not dissociate from the DNA polymerase an accompanying contaminant, which was identified by MS as *E. coli* RNA polymerase (Tables 2 and 3). Considering that the concentration of this partially purified αDr cannot be quantified, we used this enzyme preparation to perform qualitative assays, the aim of which was to confirm what we observed using refolded αDr (see below).

**Table 1:** Peptides of αDr identified by MS Identification by MS of partially purified *D. radiodurans* DnaE polymerase.

Peptide	Observed *M*_r_ (Da)	Theoretical *M*_r_ (Da)	Sequence
240–254	1597.8406	1597.8311	SDATAHETLLAIQTK.A
359–370	1201.5936	1201.5938	SLAELGEADAAR
525–539	1847.9742	1847.9669	ITNLDPLEFELLFER
671–681	1315.6844	1315.6806	EELTNLVPVMR
696–704	972.5504	972.5491	SVEDIGLIK
1035–1044	1055.4694	1055.4672	SGAFDAFGER
1089–1099	1236.6036	1236.5986	SSIAPYSDLER
1105–1123	2118.0931	2118.0858	EALGLYISGHPLEQHEGLR

**Table 2:** Peptides of *E. coli* RNA polymerase β subunit identified by MS Identification by MS of *E. coli* RNA polymerase β subunit, the presence of which was detected as contaminant of *D. radiodurans* DnaE polymerase, overexpressed in soluble form and subjected to four consecutive purification steps.

Peptide	Observed *M*_r_ (Da)	Theoretical *M*_r_ (Da)
38–54	1968.9212	1968.9217
75–88	1688.8186	1688.8192
89–97	962.5186	962.5185
119–143	2858.3134	2858.3103
144–151	950.5662	950.5661
152–161	1097.5022	1097.5030
181–191	1339.6074	1339.6085
212–227	1943.9902	1943.9880
237–245	1113.5850	1113.5852
246–260	1606.7953	1606.7951
248–260	1337.6102	1337.6099
284–295	1329.7544	1329.7544
300–324	2799.3247	2799.3194
332–352	2489.2581	2489.2550
333–352	2333.1547	2333.1539
360–368	1062.6072	1062.6073
379–402	2764.2994	2764.2980
408–422	1629.8935	1629.8937
412–422	1160.5920	1160.5925
423–430	947.4632	947.4634
423–431	1075.5598	1075.5583
440–452	1494.7174	1494.7175
455–465	1282.5612	1282.5612
479–503	2672.3752	2672.3765
504–527	2783.2901	2783.2861
530–540	1040.5984	1040.5978
648–678	3463.6207	3463.6202
707–719	1186.6558	1186.6558
721–731	1149.5776	1149.5778
759–779	2448.0817	2448.0832
780–801	2244.0726	2244.0692
802–821	2373.1138	2373.1100
828–841	1673.8558	1673.8559
845–864	2023.0462	2023.0473
865–886	2204.1576	2204.1576
891–900	1130.5448	1130.5455
945–954	1202.6218	1202.6216
959–974	1818.9340	1818.9363
977–988	1141.6342	1141.6343
997–1007	1331.6616	1331.6609
997–1022	3161.5414	3161.5404
1008–1022	1847.8900	1847.8901
1036–1048	1325.7190	1325.7191
1107–1122	1725.8908	1725.8906
1148–1156	978.4770	978.4771
1159–1171	1542.6876	1542.6872
1179–1191	1318.6586	1318.6591
1201–1211	1155.6244	1155.6248
1217–1234	2164.0345	2164.0333
1247–1262	1621.8302	1621.8312
1247–1269	2366.2048	2366.1979
1307–1328	2484.1765	2484.1777
1332–1342	1230.5980	1230.5979

**Table 3:** Peptides of *E. coli* RNA polymerase α subunit identified by MS Identification by MS of *E. coli* RNA polymerase α subunit, the presence of which was detected as contaminant of *D. radiodurans* DnaE polymerase, overexpressed in soluble form and subjected to four consecutive purification steps.

Peptide	Observed *M*_r_ (Da)	Theoretical *M*_r_ (Da)
1–12	1407.7180	1407.7180
13–25	1425.7462	1425.7464
26–33	955.5338	955.5338
34–44	1141.5990	1141.5992
46–71	2863.3981	2863.3983
72–86	1724.9572	1724.9560
92–104	1455.8317	1455.8297
96–104	1043.5864	1043.5863
105–143	4198.0437	4198.0423
159–170	1436.7001	1436.7008
171–182	1420.7020	1420.7020
183–191	1005.5252	1005.5243
201–218	2029.0038	2029.0037
219–235	1915.0528	1915.0527
220–235	1758.9514	1758.9516
244–265	2622.3904	2622.3905
272–284	1483.7797	1483.7783
285–297	1440.8191	1440.8188
299–310	1330.7456	1330.7456
318–329	1340.6236	1340.6248

### Refolding and purification of *D. radiodurans* DnaE polymerase from inclusion bodies

To pursue the isolation of highly purified αDr, devoid of *E. coli* RNA polymerase, we decided to attempt the refolding of the enzyme from inclusion bodies. The induction for 15 h at 37°C of *E. coli* TOP10/pBAD-αDr yielded 0.9 g (wet weight) of inclusion bodies per litre of culture. Upon solubilization with urea (6M), and four consecutive dialysis steps performed as described by Brown et al. [52] for yeast DNA polymerase δ, we finally obtained 27 mg of soluble proteins per g of inclusion bodies, among which αDr was highly abundant. This refolded sample was then subjected to Cibacron Blue and HiTrap Heparin affinity chromatography (Supplementary Figure S2). With both chromatographic supports, a consistent amount of αDr was lost with the flow-through, most likely containing improperly refolded enzyme. From 27 mg of dialysed proteins, we were able to recover 3.6 mg of refolded and purified αDr.

### DNA polymerase activity of refolded αDr and αEc

We compared the catalytic performances of refolded αDr with those of the well-known αEc. To this aim, we first assayed the DNA polymerase activity of both enzymes at the expense of a DNA 40mer template annealed to a 15mer primer, the extension of which exclusively depends on dTTP (Figure 1). The extension of DNA was monitored by our previously described enzyme-coupled assay (PPX assay, [48]), which relies on (Scheme 1): (i) inorganic PPase, the action of which releases P_i_ at the expense of the PP_i_ generated by a DNA Pol; (ii) PNPase, which in the presence of inosine and P_i_, catalyses the release of ribose-1-phosphate and hypoxanthine and (iii) XOD, finally converting hypoxanthine to uric acid, which is conveniently detectable at 293 nm [49]. Under these conditions, the activity of αDr was found to be approximately 90 times lower when compared with that of the *E. coli* enzyme (0.19 and 17 nM/s respectively, Figures 2A and 2B, and Supplementary Figures S3A and S3B). However, it was also observed that αDr is significantly stimulated by ionic strength, its DNA polymerase activity being approximately 4-fold higher in the presence of 200 mM NaCl or KCl (Figure 2A, and Supplementary Figure S3A). On the contrary, αEc was dramatically inhibited, i.e. 30-fold, by 200 mM KCl (Figure 2B, and Supplementary Figure S3B). Therefore, under these conditions αDr performs slightly better than its *E. coli* homologue. Moreover, when calf-thymus activated DNA was used as substrate, and all the four dNTPs were present in reaction mixtures, comparable activities were observed in the presence of αDr or αEc (0.25 and 0.3 nM/s respectively, Figure 2C, and Supplementary Figure S3C). It was previously reported that *D. radiodurans* DNA Pols I and X are positively affected by Mn^2+^ [42,44]. Accordingly, we assayed αDr in the presence of manganese, the 40mer dsDNA and dTTP. Surprisingly, a strong activation of αDr was observed, yielding an activity equal to 5.5 nM/s (Supplementary Figure S3D), whereas a small effect, if any, was detected in the presence of αEc under the same conditions (results not shown).

**Scheme 1:** Reaction paths leading to the generation of uric acid at the expense of P_i_ and inosine (upper row), and to the oxidation of β-NADH from ADP and PEP (lower row). Although the determination of uric acid can be used to assay both DNA polymerase and RecA activity, the evaluation of β-NADH oxidation is useful to specifically assay RecA in the presence of concomitant DNA polymerase activity.

**Figure 1:** Cartoon and sequences of the different DNAs used in the present study.

**Figure 2:** DNA polymerase activities detected with αDr and αEc at the expense of different DNAs. All the activity values are expressed as the increase in PP_i_ concentration (nM) per unit time (s) (**A**) Elongation rate of 40mer dsDNA by 34 nM αDr under conditions of low ionic strength (Control, dark red bar) or in the presence of 200 mM NaCl (blue bar) or KCl (pink bar). (**B**) Extension rate of 40mer dsDNA by 33 nM αEc under conditions of low ionic strength (Control, dark red bar) or in the presence of 200 mM NaCl (blue bar). (**C**) Rate of activated calf thymus DNA elongation catalysed by 34 nM αDr (green bar) or by 33 nM αEc (orange bar).

### A continuous assay for recombination-dependent DNA polymerase activity

We thought it of interest to assay the activity of αDr and αEc under conditions requiring recombination to generate a dsDNA substrate. Accordingly, we designed three oligodeoxynucleotides, two of which to be annealed into a linear 48mer dsDNA, and the third to be used as 60mer ssDNA in the assay (Figure 1). By this means, DNA polymerase activity should not be observed at the expense of dTTP, unless a previous recombination step between the 48mer dsDNA and the 60mer ssDNA occurs, generating a primer contiguous to a polyA template (Figure 1). As a first test, we assayed the binding efficiency of *E. coli* RecA to the DNAs to be recombined. To this aim, we took advantage of our PPX assay, useful to detect the RecA ATPase activity triggered by the association of this enzyme to DNA. In agreement with previous observations, we detected ATP hydrolysis coupled to the binding of RecA to ssDNA, whereas dsDNA was found to be a poor substrate (Figure 3A). We then assayed the RecA-dependence of αEc polymerase activity, using both 48mer dsDNA and 60mer ssDNA, in the presence of different dNTPs. As shown in Figures 3(B) and 3(C), only in the presence of dTTP does αEc feature RecA-dependent polymerase activity, whereas the addition of dGTP to reaction mixtures triggers the extension of DNA independently of the recombinase. Therefore, to determine recombination-dependent DNA polymerase activity, we decided to use reaction mixtures containing dsDNA, ssDNA, dTTP, RecA and ATP. In addition, we designed an assay for the simultaneous detection of the ATPase activity of RecA and the DNA polymerase activity of αEc or αDr. Our PPX assay does not indeed discriminate between DNA Pol activity and the ATPase activity of RecA. However, we thought that an additional reaction path could be coupled to RecA, i.e. the regeneration of ATP catalysed by PK at the expense of PEP, and the reduction of pyruvate to lactate by LDH, in the presence of β-NADH (Scheme 1). Using this strategy, the activity of RecA could be monitored by quantifying the consumption of β-NADH, and DNA Pol activity would be identified estimating the amount of P_i_ linked to PP_i_ hydrolysis by PPase. It should also be mentioned that the two molar absorption coefficients of β-NADH and uric acid are 6200 and 12600 M^−1^ · cm^−1^ respectively. As shown in Figure 4(A), when the absorption spectrum of a solution containing ssDNA, RecA, ATP, inosine, PNPase, XOD, PEP, β-NADH, PK and LDH was recorded as a function of time, the band of uric acid at 293 nm did progressively increase, and the band of β-NADH did concomitantly decrease, indicating the release by RecA of P_i_ from ATP. Moreover, if the absorbance values at 293 and at 340 nm are both considered as a function of time, the kinetics of RecA activity can be reliably quantified (Figure 4B). As a further test of our continuous assay for recombination-dependent DNA polymerase activity, denominated here as PPX-PL assay, we recorded absorption spectra of solutions containing a complete reaction mixture, i.e. dsDNA, ssDNA, dTTP, αEC, inosine, PPase, PNPase, XOD, RecA, ATP, PEP, β-NADH, PK and LDH. Under these conditions, the increase in absorption at 293 nm was more than twice the absorbance decrease at 340 nm, indicating the presence of DNA Pol activity triggered by the recombination of dsDNA and ssDNA (Figure 4C). Moreover, when the first minutes of the reaction are analysed in detail, it can be observed that recombination occurs first, and then DNA Pol activity takes place (Figure 4D).

**Figure 3:** ATPase activity of *E. coli* RecA and assays of αEc DNA extension activity (**A**) The release of P_i_ from ATP catalysed by 1 μM RecA was assayed in the presence of 40mer ssDNA (green dots) or at the expense of 40mer dsDNA (blue dots). (**B**) Assay of the P_i_ released by 1 μM RecA from 1 mM ATP and of the PP_i_ generated by 33 nM αEc in the presence of 48mer dsDNA and 60mer ssDNA, 1 μM each (see Figure 1). Reaction mixtures contained inosine, PPase, PNPase and XOD as coupling enzymes. Reactions were started with dGTP and dTTP (100 μM each, green dots), dGTP (blue dots) or dTTP (red dots). (**C**) Assay of the PP_i_ generated by 33 nM αEc in the presence of 48mer dsDNA and 60mer ssDNA, 1 μM each, in the absence of RecA. Other conditions are described in (**B**).

**Figure 4:** Assays of *E. coli* RecA ATPase activity and of αEc recombination-dependent DNA elongation (**A**) Difference absorption spectra recorded 5, 15, 25 and 35 min (pink, red, blue and green lines respectively) after addition of 1 μM RecA to a reaction mixture containing 1 mM ATP, 1 μM 60mer ssDNA, inosine, PEP, β-NADH, PNPase, XOD, PK and LDH. A cuvette containing a reaction mixture devoid of RecA was used as reference. (**B**) Absorbance differences as a function of time detected at 293 nm (diamonds) and 340 nm (circles) under the conditions of Figure 1(A). (**C**) Difference absorption spectra recorded during the first 10 min after addition of 33 nM αEc to a reaction mixture containing 1 μM RecA, 1 mM ATP, 48mer dsDNA and 60mer ssDNA (1 μM each), 100 μM dTTP, inosine, PEP, β-NADH, PPase, PNPase, XOD, PK and LDH. A cuvette containing a reaction mixture devoid of RecA and αEc was used as reference. (**D**) Kinetics of PP_i_ release exerted by αEc during recombination-dependent DNA elongation (diamonds), and time course of RecA ATPase activity (circles), under the conditions of (**C**). The RecA ATPase activity was determined by quantifying the coupled oxidation of β-NADH, and the release of PP_i_ by αEc was calculated via the coupled generation of uric acid, to the total concentration of which was subtracted the concentration generated by the action of RecA.

### Recombination-dependent polymerase activity of αEc and αDr

The recombination-dependent polymerase activity of αDr was tested with the PPX-PL assay, by recording absorption spectra every 10 min after the reaction was started by the addition of RecA and αDr. As shown in Figure 5(A), αDr did efficiently catalyse the extension of the dsDNA generated by *E. coli* RecA. From Figure 5(A), it is indeed clearly visible that the amplitude of the uric acid band does promptly exceed more than twice the amplitude of the negative band related to β-NADH consumption. The corresponding Δabsorbance values at 293 and 340 nm, as a function of time, were used to calculate the concentration of total P_i_ and β-NADH oxidized (Figure 5B). From the total P_i_ concentration, we then subtracted the fraction generated by RecA (corresponding to the decrease in β-NADH concentration), and we accordingly obtained the concentration of PP_i_ released by αDr (Figure 5B). Surprisingly, αDr did perform DNA extension according to a zero-order kinetics for the first 60 min of reaction time (Figure 5C), and the magnitude of this activity was significantly higher than the DNA Pol activity observed at the expense of a dsDNA not requiring recombination to be extended (cf. Figures 2A and 6A). On the contrary, when αEc was assayed under the same conditions (Figures 5D–5F), the activity of this DNA Pol was clearly much lower than the DNA extension activity observed in the absence of RecA (cf. Figures 2B and 6A). Moreover, a clear lag was observed before the DNA Pol activity of αEc entered zero-order kinetics (Figure 5F), and this kinetic regime was maintained for approximately 20 min only (Figure 5F). Overall, these observations suggest that αDr is stimulated by *E. coli* RecA, and that under the conditions of the PPX-PL assay αDr is more processive than αEc. Accordingly, we wanted to test the DNA Pol activity of both αDr and αEc under conditions requiring recombination, but in the absence of both RecA and ATP (and therefore devoid of PK, PEP, LDH and β-NADH). By this means, we wanted to assay the intrinsic recombination activity, if at all, of αDr and αEc. Surprisingly again, although αEc was clearly able to catalyse the recombination and extension of DNA, albeit at a moderate rate, αDr was incapable to perform these tasks, most likely because of its inefficiency in recombination activity (Figure 6B, and Supplementary Figure S4).

**Figure 5:** Recombination-dependent DNA extension activity of αDr and αEc assayed in the presence of RecA (**A**) Difference absorption spectra recorded every 10 min after addition of 34 nM αDr to a reaction mixture containing 1 μM RecA, 1 mM ATP, 48mer dsDNA and 60mer ssDNA (1 μM each), 100 μM dTTP, inosine, PEP, β-NADH, PPase, PNPase, XOD, PK and LDH. A cuvette containing a reaction mixture devoid of RecA and αDr was used as reference. (**B**) Kinetics of total P_i_ released by the action of RecA and αDr (filled circles), of PP_i_ generated by αDr (diamonds), and of β-NADH oxidation linked to RecA action (empty circles). (**C**) Detail of the kinetics reported in (**B**), and representing the PP_i_ generated by the recombination-dependent DNA extension activity of αDr. (**D**–**F**) Recombination-dependent DNA polymerase activity of 33 nM αEc, as determined under the same conditions of (A)–(C).

**Figure 6:** Recombinase action of RecA and recombination-dependent DNA extension activity of αDr and αEc assayed in the presence or in the absence of RecA The activity values of RecA are expressed as the increase in phosphate concentration (nM), generated at the expense of ATP, per unit time (s). The DNA extension activity values are expressed as the increase in PP_i_ concentration (nM) per unit time (s). (**A**) ATPase activity of RecA detected in the presence of αDr or αEc (green and blue bar respectively). The DNA polymerase activity of αDr and αEc are reported with dark green and dark blue bars respectively. Assay conditions are described in Figure 5. (**B**) Recombination-dependent DNA extension activity of αDr (green bar) and αEc (blue bar) assayed in the absence of RecA. The corresponding kinetics is reported in Supplementary Figure S4.

### Recombination-dependent polymerase activity of αDr overexpressed in soluble form

To further investigate the RecA-dependence of αDr polymerase activity, we performed recombination-dependent DNA extension assays using partially purified αDr overexpressed in soluble form. When the polymerase activity of αDr was tested using the PPX-PL assay (in the presence of RecA), we observed a significant extension, at the expense of dTTP, of the dsDNA generated by RecA (Figure 7). On the contrary, no DNA polymerase activity was detected when αDr was added to a reaction mixture devoid of RecA, and containing the two DNAs to be recombined and dTTP (Supplementary Figure S5). These observations qualitatively agree with those obtained using refolded αDr isolated and purified from inclusion bodies.

**Figure 7:** Recombination-dependent DNA extension activity of αDr (25 μg of P/ml) overexpressed in soluble form assayed in the presence of RecA (**A**) Difference absorption spectra recorded every 10 min after addition of αDr to a reaction mixture containing 1 μM RecA, 1 mM ATP, 48mer dsDNA and 60mer ssDNA (1 μM each), 100 μM dTTP, inosine, PEP, β-NADH, PPase, PNPase, XOD, PK and LDH. A cuvette containing a reaction mixture devoid of RecA and αDr was used as reference. (**B**) Kinetics of total P_i_ released by the action of RecA and αDr (filled circles), of PP_i_ generated by αDr (diamonds), and of β-NADH oxidation linked to RecA action (empty circles). (**C**) Detail of the kinetics reported in (B), and representing the PP_i_ generated by the recombination-dependent DNA extension activity of αDr (filled diamonds). As a comparison, the recombination-dependent DNA polymerase activity of 34 nM refolded αDr is also reported (empty diamonds).

## DISCUSSION

The purification of the αDr is described in the present study for the first time. Rather surprisingly, when overexpressed in soluble form, αDr featured a strong binding to the RNA polymerase of the host, i.e. *E. coli*. Accordingly, we were able to partially purify native αDr associated with *E. coli* RNA Pol, and we observed that the dissociation of this complex does not occur under different conditions, e.g. gel filtration or high concentrations of DTT (results not shown). Whether or not αDr does also feature high affinity for *D. radiodurans* RNA Pol remains to be ascertained. In the present study, we used the αDr–RNA Pol complex for qualitative activity assays only, designed to avoid any interference by RNA Pol on the observed activities. It should be indeed noted that we performed DNA Pol activity assays relying on dTTP as the unique nucleotide substrate. To obtain homogeneous αDr free of RNA Pol, we overexpressed αDr as inclusion bodies, and we were successful in the refolding and purification of the target protein.

When compared with *E. coli* DNA polymerase III α subunit (αEc), αDr showed quite different kinetic properties. Under standard conditions (5 mM MgCl_2_, 100 μM dTTP, low ionic strength) and in the presence of 1 μM 40mer template DNA, αDr was indeed found to catalyse DNA extension with much lower efficiency than αEc. Interestingly, when the ionic strength of the assay mixture was increased, the catalytic action of αDr and αEc was found to increase and decrease respectively. Moreover, the addition of Mn^2+^ to the reaction milieu triggered a strong increase in αDr activity, and did correspond to a modest, if at all, effect towards the action of αEc. It is interesting to note that γ-irradiation induces a general increase in cellular ionic strength, and that the accumulation of Mn^2+^ increases the radioresistance of *D. radiodurans* [53]. Therefore, our observations suggest that the activity of αDr is regulated by the conditions arising in cells upon exposure to γ-rays. In particular, the positive response of αDr to Mn^2+^ reported here agrees with previous studies concerning *D. radiodurans* Pol I and Pol X. It was indeed demonstrated that Mn^2+^ is essential for the activity of *D. radiodurans* Pol X [37], and is required to confer competence in DNA lesion bypass to DNA Pol I [42]. Accordingly, the DNA Pols of *D. radiodurans* share a strong dependence on manganese of their activities, suggesting a nice correlation with the high content of manganese that is usually detected in post-irradiated cells of this organism. However, it should also be considered that other DNA Pols, isolated from radiation-sensitive organisms, depend on Mn^2+^ for their activity, e.g. the human ιDNA Pol [54].

When considering that the ESDSA pathway of genome reconstitution is strictly dependent on αDr, one might expect that this DNA polymerase features intrinsic recombinase activity. However, αDr was found to be incapable of recombination-dependent DNA polymerase activity, independently of the strategy used to overexpress αDr in *E. coli* (Supplementary Figures S4 and S5). On the contrary, this activity was exclusively detected in the presence of both RecA and αDr. This is in sharp contrast with the catalytic properties of αEc, which was found competent in recombination-dependent DNA polymerase activity in the absence of RecA (Supplementary Figures S4 and S5). It should also be noted that the activity of αDr in the presence of RecA significantly exceeds the extension rate observed with a recombination-independent DNA substrate (cf. Figures 2A and 6A), suggesting an activation of αDr by RecA. This evidence agrees with the finding that genome replication in *D. radiodurans* RecA^−^ strains is slower when compared with that observed in the wild-type counterpart [36]. Conversely, deletion of RecA does not significantly affect the growth rate of *E. coli* [55]. Moreover, it was demonstrated that the overexpression of *recA* decreases the rate of replication fork progression in *E. coli* [29], presumably by inhibiting αEc replisomes [28].

We observed that the rate and the extent of ATP hydrolysis differ if αDr or αEc were present in RecA-dependent DNA extension assays. During the first 60–70 min after reactions started, we did indeed ascertain that: (i) when αDr was present, 5 μM dTTP was incorporated into DNA, and the hydrolysis of 10–15 μM ATP was concomitantly detected (Figure 8A); (ii) when αEc did catalyse the extension of DNA at the expense of 4–5 μM dTTP, RecA did hydrolyse 20–30 μM ATP (Figure 8B). These findings suggest that αDr does assist RecA in the recombination reaction, lowering the amount of ATP necessary to sustain strand exchange and, hence, DNA extension. Interestingly, the energetics of RecA-mediated recombination was finely dissected by a series of elegant studies. First, it was demonstrated that the rate of ATP hydrolysis triggered by the association of RecA with ssDNA slows down upon initiation of strand exchange with dsDNA [56]. Further, it was recognized that: (i) the binding of ATP or of ATP analogues converts RecA inactive filaments to an active state [57]; (ii) ATP hydrolysis and recombinational branch migration are concerted reactions [58]. Moreover, it was also shown that ATP hydrolysis induces a conformational transition of RecA C-terminus, and that this transition corresponds to the conversion of inactive RecA filaments into their active counterpart [59,60]. Finally, different states of RecA filaments were identified [61]. In the absence of ATP, RecA is in the O state and is competent in binding ssDNA [61]. When ATP is present, the recombinase switches to the A (activated) state, and the binding of ssDNA triggers ATP hydrolysis. The A state can be further characterized in two sub-states, denoted Ac (A closed) and Ao (A open), to indicate incompetence and competence in pairing reactions respectively [61]. The transition from the Ac to the Ao state was found to depend on Mg^2+^ concentration [62]. In the presence of a pairing substrate, RecA switches from the Ao to the P state, and this transition is paralleled by a decrease (approximately 30%) of the ATP hydrolysis rate [61]. According to these observations, we propose that αDr favours the transition from the Ao to the P state of RecA, therefore limiting the amount of ATP necessary to accomplish recombination. In particular, in the presence of αDr the ATP consumed per nucleotide incorporated in DNA was equal to approximately 2, whereas in the presence of αEc this ratio is more than double (Figure 8).

**Figure 8:** Kinetics of RecA-dependent DNA extension catalysed by αDr and αEc (**A**) Detail of Figure 5(B) showing the extension of DNA (diamonds) and the hydrolysis of ATP (filled circles) catalysed by αDr and RecA respectively, during the first 80 min after reactions started. (**B**) Detail of Figure 5(E) showing the extension of DNA (diamonds) and the hydrolysis of ATP (filled circles) catalysed by αEc and RecA respectively, during the first 80 min after reactions started. The concentration of PP_i_ as a function of time (corresponding to DNA polymerase activity) was calculated by subtracting the observed total P_i_ concentration to the fraction generated by RecA, and dividing the residuals by 2.

Overall, we have shown in the present study that some of the catalytic properties of αDr are in sharp contrast with those of αEc: (i) αDr is stimulated by high ionic strength, whereas αEc is strongly inhibited under the same conditions; (ii) similarly to other DNA Pols of *D. radiodurans*, αDr is activated by Mn^2+^, whereas αEc action is not significantly affected by manganese; (iii) contrary to αEc, αDr is activated by RecA, in the absence of which αDr is not able to catalyse recombination-dependent DNA extension. Remarkably, the actions of *E. coli* and *D. radiodurans* RecA proteins were reported to differ substantially [63,64]. Although *E. coli* RecA does indeed prefer ssDNA as substrate (as also shown here, see Figure 3), the *D. radiodurans* recombinase was reported to bind more efficiently to dsDNA. Accordingly, future work will be devoted to investigate the catalytic action of αDr in recombination-dependent DNA polymerase activity assays performed in the presence of *D. radiodurans* RecA protein.

## Abbreviations

DNA Pols: DNA polymerases
dNTP: deoxynucleoside-triphosphate
αDr: *Deinococcus radiodurans* DNA polymerase III αsubunit
αEc: *Escherichia coli* DNA Pol III
ESDSA: extensive synthesis-dependent strand annealing
LDH: lactate dehydrogenase
PEP: phosphoenolpyruvate
PK: pyruvate kinase
PNPase: purine nucleoside phosphorylase
PPase: inorganic pyrophosphatase
PPX: PPase-PNPase-XOD enzyme coupled assay
PPX-PL: PPase-PNPase-XOD-PK-LDH enzyme coupled assay
XOD: xanthine oxidase
